RETRACTED

# Analysis of the miRNA-mRNA Regulatory Network Reveals the Biomarker Genes in the Progression of Myocardial Ischemic Reperfusion

**DOI:** 10.1155/2022/2045619

**Published:** 2022-04-13

**Authors:** Nini Li, Qing Chen

**Affiliations:** Department of Cardiology, Xianyang Hospital of Yan'an University, Xianyang 712000, Shaanxi, China

## Abstract

**Objective:**

Cardiac injury induced by myocardial ischemic reperfusion (MI/R) is still an intractable question in clinical, and it has been confirmed as a major reason for the development of cardiovascular disease. Bioinformatics analysis has been widely used for revealing the pathogenic mechanism of diseases. This study attempted to identify the biomarkers and reveal the regulation mechanism of MI/R injury via bioinformatics analysis.

**Methods:**

The GSE67308 and GSE74951 were obtained from the GEO database. The datasets were analyzed with GEO2R tool, and the genes with |logFC| > 2 and *p* value <0.05 were identified as the differentially expressed genes (DEGs). The enrichment analysis of the DEGs was performed with the DAVID database and R language. Moreover, the protein-protein interaction (PPI) network of DEGs was performed with the STRING database and then visualized with Cytoscape.

**Result:**

The results showed that 195 downregulated mRNAs and 240 downregulated mRNAs were found in GSE67308, and 11 miRNAs were found in GSE7495. 152 common genes were screened in DEGs of GSE67308 and the targets of 11 miRNAs in GSE7495. Moreover, the enrichment analysis showed that the common genes were related with inflammatory response, immune response, PI3K/AKT, NF-*κ*B, and TNF pathways. Besides, mmu-miR-92a-3p and mmu-miR-27b-3p were identified as the hubs miRNAs, and TNF, IL1B, and IFG1 were screened as the key nodes.

**Conclusion:**

This study established a miRNA-mRNA network for cardiac injury induced by MI/R and provided the evidence concerning the molecular mechanism of MI/R injury, which provided some reference for MI/R treatment.

## 1. Introduction

Cardiovascular disease is a main risk of the human health in the world, and ischemia has been confirmed as a key reason leading the abnormal injury and apoptosis of cardiomyocyte [1, 2]. Myocardial ischemic reperfusion (MI/R) is an essential method for decreasing the rate of myocardial infarction of the patients induced by ischemia in clinical [3]. However, the dysfunction of the myocardial tissue induced by I/R may induce the inflammatory reactions and aberrant apoptosis of cardiomyocyte, which may finally increase the morbidity and mortality of the patients [4]. Therefore, the significant clinical problem of myocardial injury induced by I/R has been widespread concerned. At present, drug intervention serves as the major strategy for improving the I/R-mediated myocardial injury, and some drugs such as dexmedetomidine and captopril have been provided for the patients before the surgery to improve the injury of I/R [5, 6]. However, the pathogenic mechanisms remain not fully elucidated, and more biomarkers and targets are still necessary for diagnosis and drug development.

RETRACTED

Recently, the difference in the RNA profiling of the patients suffered I/R injury and normal persons has been revealed by increasing studies, and some genes including microRNA (miRNA) and messenger RNA (mRNA) have also been confirmed as the key factors which are associated with the development of the symptom [7, 8]. Microarray analysis of RNA abundance is an effective bioinformatics for research studies of bioresearch, and it has been widely used for identifying the biomarkers and drug targets of various disease range from general inflammation to difficult miscellaneous diseases [9, 10]. For MI/R, microarray analysis has also been used for screening the small molecule drugs. Hence, microarray analysis has been confirmed as a promising method for the MI/R study.

This study attempted to explore the effect of I/R surgery on the difference of the RNA profiling of mice, and the data of the RNA sequences were searched and obtained from the GEO database. Finally, the biomarkers and molecular mechanism of IR-myocardial injury were also revealed with bioinformatics methods.

## 2. Materials and Methods

### 2.1. Microarray Data Source

The datasets including GSE67308 tested on GPL7202 and GSE74951 tested on GPL21136 were downloaded from Gene Expression Omnibus database (GEO, https://www.ncbi.nlm.nih.gov/). For GSE67308, the data of GSM1644168–GSM1644171 and the data of GSM1644172–GSM1644175 were selected for next analysis. For GSE74951, the data of 6 sham mice groups and 9 IR mice group were used for next analysis.

### 2.2. Identification of Differentially Expressed Genes

GSE67308 and GSE74951 were analyzed with GEO2R online tool of the GEO database, and the matrix file of the genes was obtained for subsequent analysis. Moreover, the genes with |logFC| > 2 and *p* < 0.05 were selected as the differentially expressed genes (DEGs).

### 2.3. Gene Ontology Enrichment Analysis

Gene ontology enrichment analysis was performed for investigating the functions of DEGs in GSE67308 and GSE74951. Briefly, ENTREZIDs of DEGs in GSE67308 were obtained from the DAVID database (https://david.ncifcrf.gov/). After that, the packages including topGO, clusterProfiler, and org.Mm.eg.db of R language were performed to search the related functional modules of ENTREZIDs. Finally, modules with *p* value < 0.05 were visualized by R language. For GSE74951, the target of miRNAs with |logFC| > 2 and *p* value < 0.05 were obtained from miRWalk (https://miRWalk.umm.uni-heidelberg.de/). After that, the potential targets were used for GO enrichment analysis.

RETRACTED

### 2.4. Kyoto Encyclopedia of Genes and Genomes Enrichment Analysis

Kyoto Encyclopedia of Genes and Genomes (KEGG) enrichment analysis was performed to observe the related pathways of DEGs in GSE67308 and GSE74951. Simply, DEGs of GSE67308 were enriched by the online tool of DAVID database, and then, pathway modules with *p* value <0.05 were visualized with ggplot2 of R language. For GSE74951, the targets of miRNAs with |logFC| > 2 and *p* value<0.05 were selected as the potential targets and then used for KEGG enrichment analysis.

### 2.5. Network Analysis

The protein-protein interaction (PPI) network analysis was performed to select the key node genes in GSE67308 and GSE74951; DEGs of GSE67308 and the targets of GSE74951 were analyzed with STRING (https://www.string-db.org/). After that, the key nodes of the datasets were visualized with Cytoscape software. For the miRNA-mRNA network, the common genes of DEGs in GSE67308 and the targets of GSE74951 were visualized with Cytoscape.

## 3. Results

### 3.1. Identification of DEGs

The datasets including GSE67308 and GSE74951 were used to observe the effect of I/R surgery on the profiling of mRNA and miRNA of the mice. The results showed that 195 downregulated mRNAs and 240 downregulated mRNAs were found in GSE67308, and 11 miRNAs including mmu-miR-363-3p, mmu-miR-375, mmu-miR-92a-3p, mmu-miR-27b-3p, mmu-miR-27a-3p, mmu-mir-374a-5p, mmu-mir-15b-5p, mmu-miR-34a-5p, mmu-miR-370-3p, mmu-miR-30a-5p, and mmu-miR-146a-5p were found in GSE74951 (Figures 1(a)–1(c)). Moreover, 152 common genes were found in GSE67308 and the potential targets of GSE74951 (Figure 1(d)).

### 3.2. Functional Modules of DEGs

To investigate the related functions in the progression of MI/R, DEGs in GSE67308 and targets in GSE74951 were enriched by GO analysis. The results showed that 509 modules were related with DEGs of GSE67308, and DEGs were involved in the modules of inflammatory and immune regulation including positive regulation of cytokine production, leukocyte migration, cytokine-mediated signaling pathway, regulation of inflammatory response, regulation of the immune effector process, and so on (Figure 2(a)). Moreover, it was found that the common genes of DEGs in GSE67308 and targets of the miRNAs in GSE74951 were associated with positive regulation of cytokine production, positive regulation of response to external stimulus, cytokine-mediated signaling pathway, regulation of inflammatory response, production of molecular mediator of immune response, and so on (Figure 2(b)).

RETRACTED

### 3.3. Signaling Pathways Analysis of DEGs

To reveal the pathogenic mechanism of MI/R, KEGG enrichment was performed to analyze the related pathways of DEGs in GSE67308. The results showed that DEGs in GSE67308 were related with the TNF signaling pathway, cytokine-cytokine receptor interaction, NF-*κ*B signaling pathway, PI3K-Akt signaling pathway, toll-like receptor signaling pathway, and so on (Figure 3(a)). Moreover, the common genes of DEGs in GSE67308 and the targets of miRNAs in GSE74951 were related with the TNF signaling pathway, cytokine-cytokine receptor interaction, PI3K-Akt signaling pathway, NF-kappa B signaling pathway, MAPK signaling pathway, toll-like receptor signaling pathway, and so on (Figure 3(b)).

### 3.4. Protein-Protein Interaction Network Analysis

To illustrate the molecular mechanism of MI/R, DEGs of the datasets were analyzed with the STRING database. The results showed that three clusters were found in GSE67308, including cluster 1 with 64 nodes and 2156 edges, cluster 2 with 13 nodes and 48 edges, and cluster 3 with 4 nodes and 12 edges. For GSE67308, three clusters include cluster 1 with 9 nodes and 38 edges, cluster 2 with 8 nodes and 30 edges, and cluster 3 with 10 nodes and 32 edges (Figures 4(a)–4(c)). For GSE67308, STAT1, IL1B, CCL2, TNF, TLR2, CXCL10, IL6, MMP9, CCL4, CXCL 19, CXCL1, CD274, and CXCL2 were selected as the key nodes. For common genes, TNF, IL1B, and IFG1 were selected as the key nodes (Figures 4(d) and 4(e)).

### 3.5. miRNA-mRNA Network Analysis

To reveal the miRNA-mRNA interaction mechanism of MI/R, the common genes of DEGs in GSE67308 and the targets of miRNAs with |logFC| > 2 and *p* < 0.05 in GSE74951 were used for miRNA-mRNA network analysis. The results showed that 11 miRNAs and 71 genes with negative correlation of miRNAs had potential connection (Figure 5).

## 4. Discussion

Myocardial injury induced by ischemic reperfusion, one of the most dangerous diseases in the world, seriously threatens the health of senile patients, while even with current therapeutic strategies, the prognosis of the patients remains unsatisfactory [11, 12]. This study investigated the difference of mRNA profiling in MI/R and normal samples in the GEO database and analyzed the differentially expressed genes (DEGs) in the pathological samples of the patients and revealed the related pathogenic pathways and molecular interaction network via bioinformatics methods.

Myocardial ischemic reperfusion (MI/R) can promote the inflammatory reactions and mediate abnormal apoptosis of cardiomyocytes and finally induce the injury or necrosis of myocardial tissues [13]. Moreover, MI/R can also induce the significant change in gene profiling in the damaged region of the patients. Several studies have indicated that the RNA profiling in the tissues suffered with MI/R of the patients exhibits a remarkably difference with the noninjury tissues, and the similar phenomena have also been found in mice models [14, 15]. In this study, the disorder in mRNA and miRNAs profiling was also found in the mice treated with MI/R surgery via the excavating the database, and 195 downregulated mRNAs and 240 downregulated mRNAs were found in GSE67308. MicroRNA plays an important role in multiple metabolism activities of cells, and disorder of miRNAs level is major reason for formation and development of some diseases [16]. For MI/R injury, Makkos et al. indicated miRNAs in pathological samples of exhibited obvious disorder, and some miRNAs can influence the progression of MI/R injury via involving of redox signaling [17]. In this study, 11 miRNAs included were found in GSE74951. miRNA is characterized with blocking the translation of proteins by targeting the 3′-UTR of the related mRNAs. This study also investigated the targets of 11 miRNAs by the miRNA target database and found that 152 genes were also confirmed as DEGs in GSE67308. miR-363-3p has been identified as the diagnostic biomarker for MI/R injury, and upregulated miR-15b-5p, miR-34a-5p, and miR-146a-5p have been also confirmed to play promoters roles in the progression of MI/R injury [18–20]. Moreover, miR-92a-3p and miR-27b-3p have been confirmed to have connection with I/R injury or myocardial injury. The study has indicated that inhibited miR-92a-3p could effectively reduce the renal injury-associated atherosclerosis [21]. The study has indicated that miR-27b-3p could inhibit the activation of macrophages to inhibit the progression of the chronic liver injury [22]. However, in this study, upregulated miR-27b-3p was found in mice treated with MI/R surgery. Thus, those observations suggest miR-92a-3p and miR-27b-3p as the new biomarkers which may involve the progression MI/R injury via regulating the levels of the proteins.

RETRACTED

MI/R can mediate the succinate dehydrogenase activity which may promote the rapid oxidation of succinate and then induce the disorder of reactive oxygen species by reverse electron transport at mitochondrial complex I [23]. Impaired mitochondrial respiratory chain function has been confirmed as a major reason leading the cellular inflammatory reactions [24]. Increasing studies have proved that MI/R injury is related with the inflammatory reactions and immune regulations, and improving the inflammatory reaction could effectively inhibit the progression of MI/R injury. In this study, it was found that DEGs in GSE67308 were related with some cellular functional modules including the positive regulation of cytokine production, leukocyte migration, cytokine-mediated signaling pathway, regulation of inflammatory response, and regulation of the immune effector process. Thus, those proofs suggest that the inflammatory reactions and immune regulation are key events of MI/R injury. Function dysfunction induced by the change of the RNA level is associated with the dysfunction of signaling pathways in cells. Some pathways, such as STAT3, MAPK, and so on, have been confirmed as the axes which play crucial roles in MI/R-mediated injury [25]. This study found that some DEGs in GSE67308 were related with TNF, toll-like receptor, PI3K/AKT, NF-*κ*B, chemokine signaling pathway, and so on, and the common genes of DEGs in GSE67308 and the targets of miRNAs GSE74951 also had connection with PI3K/AKT, NF-*κ*B, and TNF pathways. The PI3K/AKT pathway serves as a classical avenue for cell survival and proliferation, and inhibited NF-*κ*B, TNF, and toll-like receptor pathways have been also found to alleviate the MI/R injury [26]. Thus, the targeted therapy via regulating the related pathways has been proved as a promising strategy for the treatment of MI/R-mediated injury.

In this study, the genes including STAT1, IL1B, CCL2, TNF, TLR2, CXCL10, IL6, MMP9, CCL4, CXCL19, CXCL1, CD274, and CXCL2 were selected as the key nodes. For common genes, TNF, IL1B, and IFG1 were selected as the key nodes. TNF and IL-1*β* can induce the inflammation to enhance the progression of MI/R [27, 28]. According to the abundance of the genes, IFG1 was identified as a target of mmu-miR-27b-3p. The study has indicated that IFG1 can reduce MI/R injury via activating the PI3K/AKT pathway [29]. Moreover, Chen et al. indicated that upregulated miR-27b-3p could inhibit the progression of breast cancer via targeting the PI3K/AKT pathway [30].

## 5. Conclusion

This study suggests mmu-miR-92a-3p, mmu-miR-27b-3p, and mmu-miR-370-3p as the biomarkers for MI/R injury, and mmu-miR-27b-3p promotes the progression of MI/R injury via targeting IFG1.

## Figures and Tables

**Figure 1:** The differentially expressed genes (DEGs) in GSE67308 and GSE74951. (a) Volcano plots of DEGs in GSE67308. (b) The heat maps of DEGs in GSE67308. (c) The heat maps of DEGs in GSE74951. (d) Venn diagram of DEGs in GSE67308 and the targets of miRNAs in GSE74951.

**Figure 2:** The modular functions of DEGs. (a) Module gene GO enrichment analysis of DEGs in GSE67308. (b) Module gene GO enrichment analysis of common genes of DEGs in GSE67308 and the targets of miRNAs in GSE74951.

RETRACTED

**Figure 3:** The related pathways of DEGs. (a) KEGG enrichment analysis of DEGs in GSE67308. (b) Module gene GO enrichment analysis of common genes of DEGs in GSE67308 and the targets of miRNAs in GSE74951.

**Figure 4:** The PPI network of DEGs. (a)–(c) The PPI network of DEGs in GSE67308. (d)–(f) The PPI network of the common genes of DEGs in GSE67308 and the targets of miRNAs in GSE74951.

**Figure 5:** The miRNA-mRNA network of DEGs in GSE34670.

## Data Availability

The data used to support the findings of this study are available from the corresponding author upon request.
